This article has been retracted.

# The intervention of classical and molecular breeding approaches to enhance flooding stress tolerance in soybean – An review

**DOI:** 10.3389/fpls.2022.1085368

**Published:** 2022-12-23

**Authors:** Guan Yijun, Xie Zhiming, Guan Jianing, Zhao Qian, Adnan Rasheed, Muhammad Iftikhar Hussain, Iftikhar Ali, Zhang Shuheng, Muhammad Umair Hassan, Mohamed Hashem, Yasser S. Mostafa, Yueqiang Wang, Liang Chen, Wang Xiaoxue, Wei Jian

**Affiliations:** ^1^ College of Life Sciences, Northwest Agricultural and Forestry University, Yangling, Shanxi, China; ^2^ College of Life Sciences, Baicheng Normal University, Baicheng, Jilin, China; ^3^ Rice Research Institute, Shenyang Agricultural University, Shenyang, China; ^4^ Changchun Normal University, College of Life Sciences, Changchun, China; ^5^ Jilin Changfa Modern Agricultural Science and Technology Group Co., Ltd., Changchun, China; ^6^ Plant Biology and Soil Science Department, Universidade de Vigo, Vigo, Spain; ^7^ State Key Laboratory of Molecular Development Biology, Institute of Genetics and Developmental Biology, Chinese Academy of Sciences (CAS), Beijing, China; ^8^ College of Agronomy, Jilin Agricultural University, Changchun, Jilin, China; ^9^ Research Center on Ecological Sciences , Jiangxi Agricultural University, Nanchang, China; ^10^ Department of Biology, College of Science, King Khalid University, Abha, Saudi Arabia; ^11^ Botany and Microbiology Department, Faculty of Science, Asiut University, Assiut, Egypt; ^12^ Jilin Academy of Agricultural Sciences and National Engineering Research Center for Soybean, Changchun, China

**Keywords:** soybean, flooding, tolerance, QTL, CRISPR/Ca9, omics

## Abstract

Abiotic stresses and climate changes cause severe loss of yield and quality of crops and reduce the production area worldwide. Flooding stress curtails soybean growth, yield, and quality and ultimately threatens the global food supply chain. Flooding tolerance is a multigenic trait. Tremendous research in molecular breeding explored the potential genomic regions governing flood tolerance in soybean. The most robust way to develop flooding tolerance in soybean is by using molecular methods, including quantitative trait loci (QTL) mapping, identification of transcriptomes, transcription factor analysis, CRISPR/Cas9, and to some extent, genome-wide association studies (GWAS), and multi-omics techniques. These powerful molecular tools have deepened our knowledge about the molecular mechanism of flooding stress tolerance. Besides all this, using conventional breeding methods (hybridization, introduction, and backcrossing) and other agronomic practices is also helpful in combating the rising flooding threats to the soybean crop. The current review aims to summarize recent advancements in breeding flood-tolerant soybean, mainly by using molecular and conventional tools and their prospects. This updated picture will be a treasure trove for future researchers to comprehend the foundation of flooding tolerance in soybean and cover the given research gaps to develop tolerant soybean cultivars able to sustain growth under extreme climatic changes.

## Introduction

Abiotic stresses continuously challenge our ability to increase crop yield under the extreme condition of climate change (Marli, 2021; Kairam and Sran, 2022). Climate changes increase the frequency of rainfall every year. Results showed a 30% increase in rainfall by 2030 (Zhou et al., 2021). Flooding is the second most deadly abiotic stress caused by heavy rainfall (Ye et al., 2018), which caused tens of billions of dollars of direct economic loss (Merz et al., 2021). It has caused a loss of around 3.7 billion dollars in agriculture in 2019 across the United States of America (USA) (Duffin, 2020). Generally, flood stress is categorized into two types, submergence and waterlogging, depending on the water depth (Fukao et al., 2019). Waterlogging is the form where water stays on the soil surface and plant roots are enclosed by water, whereas in submergence whole plant moderately or fully dips in water (Setter and Waters, 2003).

Flooding stress greatly affected the yield of major crops comprising soybean (Jo et al., 2022), rice (Kumar et al., 2021), and wheat (Winkel et al., 2017). Soybean is a significant legume crop grown worldwide for food, production of biofuel, and various other products due to its oil and protein contents (Valliyodan et al., 2017; Yuhong et al., 2021; Rasheed et al., 2022). Flooding stress reduces relative water content, chlorophyll contents, stomatal conductance, and carotenoid contents, as well as the activity of antioxidant enzymes in plants (Yang et al., 2011). Flooding stress decreases soybean growth and yield (Githiri et al., 2006) (**Figure 1**). Flooding stress reduced the biochemical contents of soybean, including linoleic acid and linolenic acid (VanToai et al., 2012).

**Figure 1:** Flood stress affects soybean seeds germination, seed size, seed number, seedling growth, stomatal conductance, root biomass, and photosynthesis rate, depletes protein and sugar contents, induces chlorosis and ROS, and reduces antioxidant enzyme activity. This Figure is created with Biorender.com.

The flooding tolerance mechanism is essential for agricultural sustainability. Tolerance mechanisms in soybean are not fully clarified because of the limitations in soybean germplasms (Wang and Komatsu, 2020). The soybean plant showed different defense mechanisms to counter the flooding stress, including hormonal regulation, genes, transcriptomes, proteins, and scavenging of reactive oxygen species (ROS) (Komatsu et al., 2015; Wang and Komatsu, 2020; Komatsu et al., 2021). Conventional practices like breeding methods, fertilizers, and hormones can mitigate soybean growth under flood stress (Mutava et al., 2015; Kaur et al., 2017), but they do not provide a long-term solution and are often costly and emphasizes the search for more reliable ways.

QTL mapping has been widely used to unlock the novel QTL contributing to flooding tolerance in soybean. Various QTL were identified using different mapping populations to accelerate marker-assisted selection programs (Dhungana et al., 2021b; Zhang et al., 2022). Genome-wise association studies (GWAS) have identified new genes for soybean response to flood stress (Sharmin et al., 2021). In fact application of GWAS is a powerful alternative to genes/QTL identification to strengthen the tolerance mechanism in soybean as proven by the study of Yu et al. (2019)

TFs have a significant function in the improvement of flood tolerance in soybean. Earlier studies showed the identification of potential root-related TFs accountable for controlling flooding tolerance in soybean; however, different TFs families needed to be explored for their possible role under flood stress (Valliyodan et al., 2014). Proteomics and omics (transcriptome) techniques have been employed to explore the proteins’ role in protecting soybean growth under flood stress; however, the role of several genes/proteins remained unknown, which should be studied to increase our understanding of soybean defense mechanisms under flood stress (Lin et al., 2019). Though diverse studies have been conducted, the flooding tolerance mechanism is not fully exposed. This review offered a comprehensive summary of use of influential molecular frontiers, their success stories, gaps, and upcoming research potentials.

## Effects of flooding stress on soybean

Flooding stress reduced soybean shoot growth and leaf size and caused a nutritional imbalance (Mutava et al., 2015; Hasanuzzaman et al., 2017). Flooding stress induced chlorosis, necrosis, reduced photosynthesis rate, reduced growth, decreased nitrogen fixation and plant death during vegetative and reproductive phases (Cho et al., 2006; Hasanuzzaman et al., 2016). The activity of phytohormones is largely affected by flooding stress. These phytohormones are critical for soybean growth and development. A recent study showed that flooding stress distressed the balance between GA and ABA during seed germination in soybean. Flooding stress also promoted the anaerobic condition, ethanol accumulation, a decrease in sugar contents, and increased cell conductivity in soybean (Zhou et al., 2021). Flood stress also affects the biomolecules in soybean (Oh and Komatsu, 2015). Flood stress reduced the protein concentration and deactivated APX in submerged soybean seedlings compared to the control, as Damanik et al. (2016) studied earlier. Sathi et al. (2022) observed that flooding stress increased the mortality rate and electrolyte leakage in soybean. The plant showed a delayed flowing pattern and maturity compared to control conditions (Sathi et al., 2022). Flood stress decreases the rate of respiration in roots (Wegner, 2010), and causes a decline in energy resources, loss of carbon, and deposition of noxious compounds, mainly lactate (Tamang et al., 2014). ROS-induced oxidative stress is accountable for the inhibition of antioxidant enzyme activity (Anjum et al., 2015).

Flooding stress reduced root growth, as studied by Smith et al. (2021), as they quantified the consequences at early growth phases. Flood stress reduced root dry weight (RDW), decreased total root length and root surfacer area, and the mark of injury varied among soybean lines. Short-term flooding reduced root extension and branches (Sakazono et al., 2014). Flooding stress induces injury in soybean seedlings and reduces their yield in field conditions (Mueller et al., 2021). Seed germination stages are widely affected by flooding stress (**Figure 1**). Flooding stress reduced soybean seed germination rate and ultimately reduced yield and quality Wu et al. (2017a) studied. Flooding can decrease soybean yield by 43% at the vegetative growth stage and 56% at the reproductive phase (Ye et al., 2018). Many investigations have been done on the effects of flood stress in soybean; however, additional investigations are required to deeply examine the effects of flood stress on nucleic acid, antioxidant enzymes, and the yield of contrasting genotypes.

## Mechanism of flooding tolerance and genetic diversity

Understanding the plant mechanisms to cope with unexpected flooding stress will be vital in developing novel flood-tolerant crop cultivars (Jia et al., 2021; Witt et al., 2022). Flooding tolerance is multigenetic trait, and different genes and pathways control this trait (De Oliveira, 2021). Plants have developed numerous approaches to cope with the adverse consequences of submergence situations (Zhao et al., 2021). The flooding mechanism in rice and soybean is well-studied. In the case of rice, the plant conserves respirable biomass to continue growing after flooding (Panda and Barik, 2021). One strategy is the quiescence plan, where plants do not extend shoots under flooding to lessen energy and carbohydrate consumption but continue to grow after stress. Sathi et al. (2022) revealed that soybean genotypes developed more adventitious roots in their stem, which helped plants thrive under water logging conditions (Sathi et al., 2022). Soybean plants develop aerenchyma tissue in roots, nodules, and hypocotyls which may ease the anoxia by enabling oxygen transport (Ploschuk et al., 2022).

Genetic breeding plays a key role in crop development which depends on genetic diversity (Sam et al., 2022). Genetic variation is a prerequisite for soybean flood breeding programs (Ratnaparkhe et al., 2022). Large genetic diversity increases the chances of a combination of desired alleles (Ratnaparkhe et al., 2022). Substantial yield loss can be prevented by introducing novel alleles into elite lines (Rhine et al., 2010; Vantoai et al, 2010; Ratnaparkhe et al., 2022). A group of 350 lines of soybean was screened for flooding tolerance during the initial reproductive stage (Cornelious et al., 2005). Numerous cultivated germplasm lines of soybean have been recognized as possible contributor of flooding tolerance. These potential lines were Archer, Misuzudaiz, PI 408105A, PI 561271, and PI 567651. Studies recognized wild soybean accessions that showed outstanding flooding tolerance and achieved better than PIs flooding. This indicates that wild soybean is an unexploited genetic reserve for breeding cultivars with enhanced of flooding tolerance by restoring alleles related to the tolerance that vanished during the taming of present genotypes (Valliyodan et al., 2017).

Maranna et al. (2021) evaluated 68 advanced lines of soybean to study their yield, early maturity, and flooding tolerance. Higher genetic variability for twelve traits was detected within and across three blocks. Selection for flooding tolerance under artificial circumstances exposed that NRC 128 was on equality to the tolerant variety, JS 97–52. Based on yield advantage, wider compliance, and flooding tolerance, NRC 128 was released for cultivation (Maranna et al., 2021). Kim et al. (2021) studied the flooding tolerance of 164 wild soybean relatives. Plants were treated with waterlogging stress for 14 days, and visual score assessment and discovery of vegetation indicators were performed 14 and 21 days after waterlogging (DAW). Besides, waterlogging-tolerant accessions displayed a 14.3%-56.3% rise in the projected area associated with vulnerability to waterlogging (Kim et al., 2021). This large genetic variation could be used to develop flooding tolerance in soybean. Wild relatives are a potential source of alleles and can be used in soybean breeding programs (Ratnaparkhe et al., 2022). Tran et al. (2021) also identified two wild soybean accessions that are highly tolerant to flooding stress, and these accessions could be used as a treasure trove for future breeding programs (Tran et al., 2021).

The use of untapped genetic diversity and the creation of novel germplasm resources would help to develop flood-tolerant soybean. Soybean wild relative (*Glycine soja*) can be an excellent source of novel alleles to help plants withstand flood stress. Wild accession identified earlier as flood-tolerant should be used in hybridization programs or can be a potential target for molecular breeding tools.

## Selection for flooding tolerance in soybean

Soybean selection for flooding tolerance is mainly phenotypic, indicating the natural variations among the population (De Oliveira et al., 2022b). With the discovery of novel breeding methods, uses of standard breeding methods are limited (Rahman et al., 2022). The screening and selection of flood-tolerant soybean cultivars have been practiced to ensure yield stability. It is significant to breed flood-tolerant soybean cultivars for seed production in areas of heavy rainfall (Sathi et al., 2022). In an earlier study, Ali et al. (2018) screened 11 soybeans cultivars against flood stress. They identified NN1138-2, M8206, and ZXD as superior flood-tolerant lines, which can serve as a valuable source of genes/alleles for future research studies (Ali et al., 2018).

Earlier, Wu et al. (2017b) evaluated 722 soybean genotypes for flooding tolerance in five years of flood screening tests. Eleven genotypes exhibited consistent flooding tolerance during 4-5 years of continual evaluations. These results showed the importance of conventional screening methods and their applications in selecting flood-tolerant soybean (Wu et al., 2017b). The effects of each breeding method are different for flood tolerance in soybean. Conventional breeding and selection practices have been widely used to screen soybean genotypes tolerant to flooding stress. Pokhrel et al. (2021) identified the soybean cultivars suitable for growing under extreme soil moisture conditions. They identified TGX 1990–94F and SBO –115 as appropriate for flood stress. These genotypes can be used directly in the hybridization program to breed high flood-stress tolerance cultivars (Pokhrel et al., 2021). A recent study showed that two wild soybean accessions were highly tolerant to submergence, and two other wild soybean accessions and 3 EMS soybean lines were also tolerant. In wet soil conditions, two accessions and ten others in the wild population were highly tolerant (Tran et al., 2021). In a later experiment, two wild soybean accessions were selected to be tolerant to flood stress at the germination phase, having a 90% higher seedling rate than control conditions. In additional studies, the tolerant lines screened could be used for the breeding program to recognize the genetic regions accountable for flooding tolerance (Tran et al., 2021). Sathi et al. (2022) identified soybean genotypes GC-840, BINAsoybean-1, BARI Soybean-5, Sohag, and BINAsoybean-2 with improved tolerance levels to flood stress and predicted the use of genotypes in areas with high rainfall (Sathi et al., 2022). Nguyen et al. (2018) screened 380 soybean accessions for flood tolerance, and eight lines exhibited a tolerant phenotype (Nguyen et al., 2018).

In another study, the effects of divergent selection approaches were studied at the F_4:5_ and F_4:6_ phases on the response to flooding tolerance and yield at the F_4:6_ stage (De Oliveira et al., 2022b). Different populations were subjected to flooding stress. The top 15% of lines were marked for assortment, except for marker-assisted selection (MAS), which was adjusted based on retrieval of chosen haplotype. Classical breeding methods have several limitations, as they are time-consuming, costly, and not very powerful to develop highly flood-tolerant cultivars due to the complexity of the trait. Backcrossing, pedigree selection, and mass selection breeding approach still need a deep investigation for their potential use in the selection of flood-tolerant soybean cultivars.

## Role of growth hormones in flood tolerance

To recognize the physiological mechanism during flood stress, diverse phytohormones were exogenously applied to soybean plants (Kim et al., 2018; Wang and Komatsu, 2022). ET is the most dominant of these hormones, which has been firmly recognized as a critical indication of flood tolerance (Zhao et al., 2021). ABA is the main stress-responsive hormone in plants. It is also known as a “stress hormone” that controls numerous responses to abiotic stresses, but its role in flood tolerance leftovers many gaps (Zhao et al., 2021). Hormonal application is a well-known agronomic approach to mitigating the toxic effects of flood stress in soybean (Kang et al., 2021; Pan et al., 2021; Tamang et al., 2021; Wang and Komatsu, 2022). Tamang et al. (2021) revealed that abscisic (ABA) acid and ethylene (ET) are candidate hormones that direct transcriptomic energy-saving developments under flood stress. Auxin may be a signaling factor differentiating submergence-specific control of the stress response in soybean (Tamang et al., 2021).

An earlier study showed that endogenous hormones (ET, GA) significantly improved the soybean response to flooding stress. Tolerant soybean lines showed higher contents of ET and gibberellic acid (GA) hormones than the sensitive line, and these hormones have a key role against flooding stress (Kim et al., 2015). Another important plant hormone is jasmonic acid (JA) (Raza et al., 2021), which controls several functions under flood stress. JA increased the activity of monodehydroascorbate reductase in soybean plant roots under flooding stress. This proposes that the number of lateral roots, and total root mass, largely donate to biophoton emission. Monodehydroascorbate controls the hydrogen peroxide level and may safeguard plants against oxidative stress (Kamal and Komatsu, 2016).

Kim et al. (2018) investigated the role of ET in mitigating the harmful effects of flood stress on soybean. Outcomes exhibited that using ETP alleviated flood stress, meaningfully enhanced the photosynthesis pigment, and enhanced the endogenous GAs contents compared to control plants (Kim et al., 2018) (**Figure 2**). GA also alleviates the adverse effects of flood stress on soybean. GA application induced the glutathione activity and condensed the resulting superoxide anion content during short-term flooding in soybean. These outcomes showed that GA plays a regulatory role in biochemical changes in soybean (Khan et al., 2018). CK also plays a key role in improving plant growth and functions under flood stress, but its role is poorly understood in crops (Islam et al., 2022). Effects of hormones under short-term and long-term flood stress should be compared in soybean. Studies on hormonal effects on biochemical pathways activity of antioxidant enzymes should be enhanced to develop an effective physiological and biochemical-based tolerance mechanism in soybean. These research gaps must be covered in future studies.

**Figure 2:** Soybean counters flooding stress by using adventitious roots and aerenchyma. Besides this gaseous hormone, ethylene (ET) causes the plant to switch to an emergency power system. Hormones mitigate plant growth under flood stress via increasing chlorophyll contents, protein, synthesis, etc. Conventional breeding methods are powerful tools for developing flood tolerance in soybean. This Figure is created with Biorender.com. (Template adapted from: Daisy Shu, PhD Postdoc, Schepens Eye Research Institute, Harvard Medical School).

## QTL identified for flood tolerance in soybean

QTL mapping is the most influential method for identifying the potential genomic areas controlling flood tolerance in soybean (Nguyen et al., 2021). The choice of the population is extremely important to recognize the genomic areas controlling flood tolerance in soybean. Recombinant inbred lines (RIL) are mostly used for QTL mapping (Cornelious et al., 2005). In the latest study, a major flood-tolerant QTL was mapped in soybean F_5_-derived RIL population made from by crossing Benning × PI 416937. Nine significant QTL were detected on chromosomes 1, 4, 5, 16, and 18. These QTL for flooding tolerance score (FTS) and survival rate (SR) were stable QTL and may be useful in the breeding of flood-tolerant genotypes of soybean (Zhang et al., 2022). Earlier, two QTL for flooding tolerance at the seedling stage were mapped in soybean and are relatively consistent in the NJRISX population (Sun et al., 2010). In another study, several QTL were mapped for soybean flood tolerance at the seedling phase. Two significant QTL were detected on chromosomes 7 and 3 under DWI in 2017 and 2018, exhibiting the highest (25.6%) and lowest (8.3%) phenotypic variance, correspondingly (Dhungana et al., 2021b). Seed water logging tolerance is critical to sustaining soybean growth and production under flood stress. Sayama et al. (2009) reported the identification of four QTL for seed flooding tolerance in soybean on chromosomes 1, 2, 3, and 4. and highlighted the physiological effects of genetic regions controlling flooding tolerance in soybean (Sayama et al., 2009). Two QTL, for flooding tolerance score (FTS) were mapped on chromosome 11 and 13 using the RIL population, and results showed that these QTL played a key role in improving flooding tolerance in soybean. QTL, on chromosome 13 was stable QTL as validated in this study (Nguyen et al., 2012). QTL detected for root development under waterlogging conditions were confirmed using near-isogenic line (NIL), NIL-9-4-5. The QTL for flooding tolerance in RIL was detected in the same region as in NIL. Results indicated that QTL, on chromone 12 controls the flooding tolerance in soybean (Nguyen et al., 2021).

Dhungana et al. (2020) imposed flood stress at the V1–V2 stage of the RIL population, and leaf chlorophyll contents were measured under control and flood conditions. A total of 20 QTL were identified on nine chromosomes. QTL, on chromosomes 9 and 10, were identified for chlorophyll content. These regions could maintain photosynthesis under flooding stress (Dhungana et al., 2020). Van Nguyen et al. (2017) detected 11 QTL for various root traits. QTL for root length development (RLD) and root surface area development (RSAD) were stable QTL between 2 years. Near-isogenic lines (NIL) were developed to validate the QTL derived from Iyodaizu (Van Nguyen et al., 2017). The QTL for root development was detected on chromosome 12 using the NIL-9-4-5 population and provided a significant role in root-based flood tolerance mechanisms in soybean. The QTL was validated using the NIL population (Dan and Tu, 2021). A QTL, was identified on chromosome 7 in the RIL populations for flood damage score (FDS) and confirmed the population flood tolerance in soybean. QTL was stable in both population (Hummer, 2018). In soybean roots plasticity and architecture also improve the flooding tolerance, and studies have identified the genetic variation associated with these traits. The main QTL, (**Table 1**) on chromosome 3, harboring tolerant allele from the exotic parent, was isolated from the NIL population, and its effects on water logging tolerance were checked in various environments. Its contribution to waterlogging tolerance was validated in many environments (Ye et al., 2018).

**Table 1:** QTL identified for flood tolerance in soybean.

Populations/parents	QTL	Chromosome	References
RIL (Benning × PI 416937)	*qFTS-1*, *qSR-5.1*	1, 5	(Zhang et al., 2022)
RIL, NIL-9-4-5 (Tachinagaha, Iyodaizu)	*qRD-12*	12	(Dan and Tu, 2021)
RIL (Danbaekkong × NTS1116)	*qSFT_7-3* and *qSFT_3-64*	7, 3	(Dhungana et al., 2021b)
RIL (Tachinagaha × Iyodaizu)	*qGR-12*	12	(Nguyen et al., 2021)
RIL (Paldalkong × NTS1116)	*qSFT_9-22*, and *qSFT_10-52 *	9, 10	(Dhungana et al., 2020)
111, 79 RIL	*qFDS-7*	7	(Hummer, 2018)
182 RIL (S99-2281 × PI 561271)	*qWT_Gm03*	3	(Ye et al., 2018)
RIL (Tachinagaha × Iyodaizu)	*Qhti-12-1*, *Qhti-12-2*	12	(Van Nguyen et al., 2017)
RIL (S99- 2281 ×PI 408105A)	*FTS-11, FTS-13*	11, 13	(Nguyen et al., 2012)
96 RILs	*Sft1*, *Sft2, Sft3*, *Sft4*	1, 2, 3, 4	(Sayama et al., 2009)
60 RIL (Misuzudaiz × Moshidou Gong 503)	*qft-6*, *qft-7*	6, 7	(Githiri et al., 2006)

All these studies showed the identified QTL controlling flooding tolerance in soybean (Nguyen et al., 2012; Nguyen et al., 2021; Zhang et al., 2022). Studies on QTL pyramiding to breed flood-tolerant soybean cultivars are limited. The effects of genomic regions on physiological and biochemical traits udder flood stress are poorly understood. In future studies, breeders should focus on developing soybean cultivars tolerant to flooding stress using MAS selection.

## GWAS-based identified QTL and genes for flood tolerance

Recognizing quantitative trait loci (QTL) and analyzing the inheritance of flooding tolerance will aid in breeding soybean genotypes tolerant to flooding stress (Wu et al., 2020). GWAS studies have recognized the mechanism of seed flooding tolerance in soybean. Many studies have identified the regions and genes associated with flooding tolerance. Novel genes and SNPs significantly contributed to soybean flood tolerance (Rohilla et al., 2020; Wang et al., 2020; Manik et al., 2022). GWAS has identified 25 and 21 quantitative trait nucleotides (QTN) linked with germination rate (GR), normal seedling rate (NSR), and electric conductivity (EC) (Yu et al., 2019). Remarkably, QTN13, on chromosome 13, has been constantly recognized as related to all three studied traits in both approaches and numerous environments. Moreover, subcellular localization exhibited that, *GmSFT* was confined in the nucleus and cell membrane. Hence, this gene was the most expected candidate gene for seed flooding tolerance in soybean (Yu et al., 2019).

A nested association mapping (NAM) population of 230 lines of RIL was developed for flooding tolerance. GWAS has identified 26 main effect QTL with 63 alleles. The best genotype was predicted to have a value of 1.924, and 33 candidate genes were identified for six biological processes (Ali et al., 2020). Wu et al. (2020) evaluated a panel of 320 soybean plant introductions (PIs) for flooding tolerance. Fourteen SNPs were recognized as linked to flooding tolerance in soybean, and five were linked with coding regions of candidate genes (Wu et al., 2020).

Soybean morphological traits, shoot length (SL), and root length (RL) have been studied for flooding tolerance. The earlier study detected the SNPs on chromosomes 1 and 5, linked to RL and SL. These novel regions regulating flooding tolerance in soybean may assist in further molecular studies (Sharmin et al., 2021). The mining of flood-tolerant genes has been the main goal of the breeders. Previously 83 genes were mined in the soybean population using bioinformatics big data mining and integration techniques. The results of 83 genes were validated using several independent databases (Soy database, GO database, and transcriptome database) and showed that these genes were superior to other genes (Lai et al., 2021). These genes/SNP provided valuable data for molecular breeding to develop flood-tolerance soybean cultivars. Data analysis indicated that GWAS had identified QTL, SNP, and genes for flooding tolerance in soybean; however, information is still insufficient and does not cover all aspects of flood tolerance. More studies must be conducted to identify the genomic regions and use them in the soybean flood breeding program (Sharmin et al., 2021). Using a more stable population (RIL) for GWAS would help uncover several novel loci/genes and trait markers associations controlling flood tolerance in soybean.

## Transcription factors analysis for flood tolerance

Root-related TFs play a key role in response to low oxygen levels under flood stress. TFs are divided into different families based on their function (Fuhrmann-Aoyagi et al., 2021). The flood-induced expression level of TFs indicates the tolerance mechanism of soybean cultivars (Fuhrmann-Aoyagi et al., 2021). Valliyodan et al. (2014) evaluated soybean cultivars PI408105A and S99-2281 to examine their response to flood stress and understand the differential gene expression. To investigate the flood response, the qRT-PCR technique was used to investigate the gene expression underlying flood tolerance by root-related TFs, known as anaerobic genes. A total of 132 genes were identified with different expressions (Valliyodan et al., 2014). Hypocotyl of soybean seedlings is also disturbed by flooding stress. Transcriptional response to flood stress in the hypocotyl of soybean seedlings has been studied. More than 6000 genes in response to flood stress in roots hypocotyl of seedlings have been identified. Transcriptional analysis showed that these genes were significantly upregulated and related to photosynthesis and cell death. This gene might protect the plant from flood-induced injury (Nanjo et al., 2011). TFs family bZIP plays a key role in responding to soybean flood stress. Expression of bZIP TF *AtAREB1* activates the cross signaling response in soybean under flood stress (**Table 2**). The expression of *AtAREB1* was enhanced by flood stress. Genetically altered soybean plants overexpressing *AtAREB1* showed improved tolerance to flooding stress (Fuhrmann-Aoyagi et al., 2021).

**Table 2:** TFs identified for flood tolerance in soybean.

TFs	Gene	Role	References
bZIP	*AtAREB1*	Enhanced cross signaling response by increasing protein content and lowering the content of hydrogen peroxide	(Fuhrmann-Aoyagi et al., 2021)
bHLH, bZIP, ERF, MYB, WRKY	22,468	Upregulated and enhanced flood tolerance	(Dhungana et al., 2021a)
bZIP	*GmbZIP1*, *GmbZIP160*	Showed transcriptional abundance in all tissues under flood stress	(Zhang et al., 2018)
WRKY	23 genes	Regulation of cell wall precursors and sugar content	(Chen et al., 2016)
NAC2	*NAC*	Expressed during initial days of flooding stress	(Valliyodan et al., 2014)

Two more bZIP TFs *GmbZIP1* and *GmbZIP160*, were detected in the soybean genome. After investigating the expression profiling of *GmbZIP* in different tissues under flood stress, it was concluded that most of these genes showed transcriptional abundance in all tissues and may play a key role in developing flood-tolerant cultivars in soybean (Zhang et al., 2018). Chen et al. (2016) identified the 3498 differently expressed genes under flood stress in soybean. These genes belong to Basic Helix-loop Helix (bHLH), WRKY, and Ethylene Response Factors (ERFs) and are involved in flood tolerance mechanisms. Changes in gene expression in sugar content can serve as an adaptive mechanism under flood stress (Chen et al., 2016). Recently, Dhungana et al. (2021a) also analyzed differentially expressed genes by RNA sequencing in leaf tissues of soybean tolerant cultivar (Paldalkong) and susceptible (NTS1116). A total of 22,468 genes were identified differently expressed in flood-stressed conditions compared to the control conditions. The number of abscisic acid-related bZIP was higher in tolerant cultivars. These identified genes could be a potential target for genetic engineering (Dhungana et al., 2021a).

## Transcriptome analysis for flooding tolerance in soybean

Transcriptome studies have identified several genes (upregulated and downregulated) for flood tolerance in soybean (Li et al., 2022). Several genes and proteins are involved in soybean response to flood stress (Chen et al., 2016). In an earlier experiment, 97 genes showed greater than 25 folds change following 12 hours of flood stress treatment (Komatsu et al., 2009). Two potential genes (*GsCNGC20-f* and *GsCNGC20-g*) were recognized from the *Glycine soja* accession (P18B), which is submergence tolerant. These findings could provide a new perspective on the molecular breeding of flood-tolerant soybean (Li et al., 2022). Very little is known about seed flooding tolerance in soybean. A total of 1563 and 1958 differentially expressed genes were recognized in tolerant and sensitive cultivars (PI342618B, NN86-4/SFS), respectively, suggesting that the former is less affected by flooding stress. Five identified genes, *Glyma.01G231200*, *Glyma.08G083300*, *Glyma.06G045400*, *Glyma.05G215900*, and *Glyma.15G015100*, demonstrated both important contradictory expression outline and nucleotide alterations, correspondingly between tolerant and sensitive (Sharmin et al., 2020). Lai et al. (2021) identified 83 significantly superior genes in soybean under flood stress (Lai et al., 2021).

RNA sequence-based transcriptome analysis is extremely popular for mining the potential genes involved in flood tolerance in soybean. Transcriptome analysis has identified a total of 31 genes, including 12, which showed identical ways of expression and were commonly altered in these plant groups under flooding stress. They were mostly accountable for RNA regulation and protein metabolism (Yin et al., 2017). Stress-responsive transcriptomes and hormonal profiling have been critically discussed previously. Tamang et al. (2021) developed a new transcriptome response analysis and revealed that ABA and ethylene responses were activated under flood stress. ABA and ethylene are applicant hormones that organize transcriptomic energy-saving processes under flood stress (Tamang et al., 2021). A miRNA comparative study was conducted to identify the different miRNAs and their stress-related genes involved in flood tolerance in soybean cultivars (Cheongj-3). A total of 247 conserved miRNAs were found, and miR319 and miR390 appeared to be linked to non-coding RNAs. These findings provided information on miRNAs and their genes in Cheongj-3 (Jhang et al., 2019). The comparative expression of genes related to flooding, including enolase (ENO), and alcohol dehydrogenase 1 (ADH1), was assessed using transcription polymerase chain reaction (RT-qPCR). Gene expression increased flood tolerance in soybean roots. The tolerant soybean cultivar (I27) showed higher expression of genes involved in energy metabolism and detoxification and indicated a flood tolerance mechanism (Casarotto et al., 2019). Two flood-tolerant genes (*Glyma.12g030900*, *Glyma.10g050300*) identified in leaf and root tissues showed higher expression in tolerant lines than in susceptible lines (Dhungana et al., 2021c). Core clock *SUB1* and *ABAR* genes mediated flood tolerance in soybean by alternate splicing. *PRR3* showed flooding-specific splicing patterns and may work with *PRR7* and *TOC1* to attain energy homeostasis under flooding circumstances (Syed et al., 2015). Besides all these factors, Khan et al. (2019) reported that ABA and nitric oxide (NO) genes could mitigate the negative effects of flood stress in soybean. The mgRNA expression of *NO overproducer1* (*NOX1*) and *ABA-receptor* (*ABAR*) were evaluated. The transcripts of NOXI were responsible for NO homeostasis during the initial phase of flood stress (Khan et al., 2019). Imran et al. (2022) also reported the NO-based modulation of soybean growth under flood stress. *GSNOR* and *NR* expression was enhanced by SNP treatments and improved the cellular SNO level, positively affecting flooding stress tolerance (Imran et al., 2022) (**Table 3**). Certain TFs families are not deeply investigated and these gaps must be covered in future studies. Further studies would facilitate identifying genes/TFs involved in the flood tolerance mechanism. Many unknown genes should be identified *via* detailed genetic analysis of the soybean genome under flood stress.

**Table 3:** Transcriptomes for flood tolerance in soybean.

Genes	Role	References
*GsCNGC20-f, GsCNGC20-g*	Enhanced calcium cascade	(Li et al., 2022)
*GSNOR, NR*	Improved the cellular SNO level	(Imran et al., 2022)
*Glyma.04g240800*	Alcohol dehydrogenases (ADH) contributed to flooding tolerance	(Lai et al., 2021)
*Glyma.12g030900, Glyma.10g050300*	Showed higher expression in tolerant lines	(Dhungana et al., 2021c)
*Glyma.01G2* *31200, Glyma.08G083300*	Enhanced seed flood tolerance in soybean	(Sharmin et al., 2020)
*NOX1*	NO homeostasis	(Khan et al., 2019)
*Glyma16g02050, Glyma17g01870*	Involved in RNA regulation and protein metabolism	(Yin et al., 2017)

## Proteomics analysis for flood tolerance

Proteins are a key element in soybean response to flooding stress (Zhong et al., 2020). The proteomics technique has extensively recognized novel proteins under flood stress in soybean (Lin et al., 2019). Khan et al. (2022) applied gel-free proteomics to investigate the soybean response to flood stress. 539 and 472 proteins were identified under control, and flood stress and 364 proteins were commonly detected in both experiments (**Table 4**). These results indicated that soybean response to flood stress by bringing biochemical changes and adopting less energy-consuming techniques (Khan et al., 2022). Likewise, a 2-day-old mutant line of soybean was exposed to flooding stress using a gel-free proteomic method. Oppositely altered proteins in abundance between the wild type and mutant line under flooding stress were related in the endoplasmic reticulum as indicated by gene-ontology categorization (Komatsu et al., 2021). Wang et al. (2021) identified 634, 1401, and 1205 proteins under control, flood, and melatonin conditions. These proteins were lined with the metabolism of proteins, RNA, and cell walls. These findings propose that factors associated with the degradation and functional positions of RNA play key roles in enhancing the effects of melatonin on soybean plants under flooding stress (Wang et al., 2021).

**Table 4:** Identified proteins for soybean response to flood stress.

Proteins	Role	References
Control 539 and flood stress 472	Biochemical changes to counter toxic effects of flood stress	(Khan et al., 2022)
Glycoproteins	Glycoproteins increased under flood stress and protected the soybean mutant line	(Komatsu et al., 2021)
634, 1401, and 1205 proteins under control, flood, and flood plus melatonin treatment	Promoted soybean growth under flood stress	(Wang et al., 2021)
Beta-amylase 5 and beta-glucosidase 31	Gene expression of beta-glucosidase 31 was upregulated	(Wang et al., 2017)
Chaperon 20, enolase, and polygalacturonase inhibit protein	These proteins increased in abundance and triggered flood tolerance	(Yin et al., 2016)
365 nuclear proteins	Increased flood tolerance in soybean	(Yin and Komatsu, 2016)
Ferritin 1, zincin-like metalloprotease, and cupin family proteins	Detoxification of ROS	(Kamal et al., 2015)
RNA binding related proteins and flood stress indicator proteins	Significantly associated with flood tolerance index	(Nanjo et al., 2014)
94 nuclear proteins	Protein synthesis and posttranslational modification	(Won Oh et al., 2014)
111 and 69 glycoproteins	Involved in glycolysis	(Mustafa and Komatsu, 2014)
U2 small nuclear ribonucleoprotein	Enhanced flood tolerance by energy conservation	(Komatsu et al., 2013)
799 proteins	Scavenging of ROS	(Komatsu et al., 2009)

Sometimes soybean plants were treated with different treatments along with flooding stress. In an experiment, two days old soybean seedling was flooded, and proteomic analysis was done using the gel-free proteomic method. The abundance of 34 nucleic proteins like histone deacetylase and U2 small nuclear ribonucleoprotein was enhanced by ABA supplement under flooding stress; however, zinc finger protein and importin alpha were reduced (Komatsu et al., 2013).

In another experiment, 146 proteins were changed in the initial flooding stage. Chaperon 20 and RNA regulation-related proteins were abundant at protein and RNA expression levels. Results showed that enolase and polygalacturonase-inhibiting proteins were abundant during the survival phases (Yin et al., 2016). Nanjo et al. (2014) evaluated the 128 soybean varieties under flood stress and conducted a proteomic analysis. RNA binding-related proteins and flood stress indicator proteins were associated with the flood tolerance index. Results showed that the flood tolerance mechanism depends on the abundance of identified proteins (Nanjo et al., 2014). Despite all of these studies, the flood tolerance mechanism in soybean is unclear. The proteome technique showed that 34 out of 799 proteins changed after 12 hours of flood stress (Komatsu et al., 2009). The growth duration of soybean seedlings is a key step to be considered during flood stress treatment. Most studies showed that 2 days old soybean seedling is suitable for flood treatment. Glycoproteins are the most significant class of stress-related proteins. Mustafa and Komatsu (2014) treated 2 days old soybean seedlings with flood stress and collected roots for proteomic analysis. A total of 111 and 69 glycoproteins were recognized without and with 2 days of flood stress. A comprehensive analysis of proteins showed that glycoproteins involved in glycolysis are activated and might be responsible for flood tolerance (Mustafa and Komatsu, 2014).

Organ-specific proteins greatly affect the soybean response to flood stress. An earlier study has identified 17 proteins, including beta-amylase five and beta-glucosidase 31, in soybean seedlings under flood stress. Gene expression of beta-glucosidase 31 was upregulated in leaves exposed to flood stress, and the expression level was correlated with protein abundance (Wang et al., 2017). The root tip is the most sensitive organ under flood stress. Hence, identifying organ-specific proteins gives a clearer understanding of soybean flood tolerance. Protein profiles specified that fermentation and protein synthesis were vital in root tips under flooding stress (Wang et al., 2016).

Analysis of soybean cotyledon provides insights into protein identification under flood stress. The 165 proteins from cotyledon were recognized under flooding stress in soybean. These results suggest that ferritin might be vital in defending plant cells against oxidative injury under flooding circumstances (Kamal et al., 2015). Nuclear proteomics analysis revealed the role of protein synthesis in the root of soybean under flood stress. Yin and Komatsu (2016) revealed that 365 nuclear proteins changed in the root tip of soybean during initial flood stress. Protein translation was suppressed during flooding stress (Yin and Komatsu, 2016). 94 nuclear proteins (**Table 4**) were identified under flooding stress. Out of 94 proteins, 19 and 75 were enhanced and decreased correspondingly. The known flooding-responsive proteins were classified, indicating that eight increased proteins altered protein synthesis and degradation of protein, whereas 34 decreased proteins were accountable for transcription and chromatin structure maintenance (Won Oh et al., 2014). All of these studies indicated the role of stress-responsive proteins in soybean (Khan et al., 2022). The role of organ-specific proteins is poorly understood and needs more studies. Future studies should focus on types of proteins and their mechanism of action especially nuclear proteins. The timing and duration of flood stress can affect the expression of proteins, which will help us alter the protein function as per requirements.

## Transgenic breeding for flood tolerance in soybean

Genetic engineering plays an important part in developing flood-tolerant genotypes in many crops and soybean (Tereshonok et al., 2010; Chiang et al., 2015; Song et al., 2018; Torti et al., 2020). Many flood-tolerant cultivars have been developed using different breeding methods (**Table 5**). The soybean genome has been characterized for its potential genes for flood tolerance. In an earlier study, Song et al. (2018) identified 61 *XTH* genes and categorized them into three subclasses based on phylogenetic analysis. Comprehensive analysis showed that most GmXTHs genes revealed organ-specific expression patterns. The expression pattern was mainly linked with ethylene and flood stress. Transgenic plants showed flood tolerance and a higher germination rate (Song et al., 2018).

**Table 5:** List of flood-tolerant cultivars of soybean.

Sr. No	Genotypes	References
1	Misuzudaizu	(Githiri et al., 2006)
2	Peking	(Sayama et al., 2009)
3	Benning	(Zhang et al., 2022)
4	Danbaekkong	(Dhungana et al., 2021b)
5	I27	(Casarotto et al., 2019)
6	Pangsakong’, ‘Geumkangkong’, and ‘Soho-kong’	(Dhungana et al., 2019)

*GsCNGC20-f* alleviated flood stress in transgenic soybean by enhancing anaerobic respiration (Li et al., 2022). Alcohol dehydrogenase transgene showed significant tolerance against stress flood stress. Flood stress response was studied in transgenic lines of soybean in which the soybean Adh (*GmAdh2*) gene was introduced under the control of a constitutive promoter. These outcomes specified that the introduced *GmAdh2* gene might have brought some change in glycolysis and alcohol fermentation and enhanced the germination of transgenic soybeans under flooding stress (Tougou et al., 2012). Recently, De Oliveira et al. (2022a) evaluated the transgenic soybean line overexpressing the *NCED* gene (2Ha11). *NCED* overexpression reduced seed weight and grain yield in the 2Ha11 line under waterlogging at the reproductive phase. These outcomes suggested that the overexpression of *NCED* activates an enhanced flooding sensitivity in soybean plants, particularly after treatment with waterlogging at the reproductive phase (De Oliveira et al., 2022a). Genetic engineered soybean could play a crucial part in the advancement of flood-tolerant soybean cultivars. Until now, available information is insufficient, and it is direly needed to conduct more studies to develop transgenic soybean to counter the toxic effects of flood stress on soybean. Use of genetic engineering to improve soybean roots growth would lead to better adaptation under flood stress as the root is the first organ disturbed by flood stress.

## CRISPR/Cas-based gene editing for flood tolerance in soybean

CRISPR/Cas9 has opened a new way of gene editing in crops (Rahman et al., 2022). Newly developed gene manipulation tools, such as CRISPR/Cas9, cemented the ways for improved genetic alteration of soybean (Rahman et al., 2022). The use of CRISPR/Cas9 systems and plans for improving its specific role is debated. CRISPR/Cas9 is an adaptive immune system in bacteria that protects them from virus attacks (Rasheed et al., 2021). CRISPR/Cas9 has two components, single-guided RNA (sgRNA) and Cas9 protein (**Figure 3**). SgRNA guides the Cas9 protein to align it to the targeted gene, and Cas9 cuts the gene and causes mutations (Rasheed et al., 2021). Non-homologous end joining (NHEJ) and homology direct repair (HDR) are used to repair the mismatched sequences in the genome (Rasheed et al., 2021). The number and variety of known CRISPR/Cas systems have considerably enlarged in recent years. The new classification comprises two classes, six types, and 33 subtypes, compared with five types and 16 subtypes previously reported. Another major innovation is the detection of many derived CRISPR/Cas9 alternatives, often related to mobile hereditary elements that lack the nucleases obligatory for interfering. There are two CRISPR/Cas9 system classes, Class 1 and Class 11 (Koonin et al., 2017).

**Figure 3:** One of the most significant and consistent ways to develop flood-tolerant soybean varieties is using molecular breeding tools. CRISPR/Cas9 is a new and influential gene manipulation tool among all molecular breeding tools. This tool can develop flood-tolerant cultivars and bring agricultural revolution. This Figure is created with Biorender.com.

Still, CRISPR/Cas9 for gene editing for flood tolerance is rarely reported (Xiao et al., 2021). Xiao et al. (2021) used CRISPR/Cas9 tool to edit the two paralog genes (*GmpPLA-IIϵ* and *GmpPLA-IIζ*), to study their modulating role in soybean response to flood stress. 112 *GmPLAs* were recognized in the soybean genome, including 78 PLA1, 29 patatin-like PLAs, and five secretory sPLA2. Segmental and Tandem duplication incidents are responsible for the extension of PLAs in the soybean genome. Some CRISPR/Cas9-generated mutant lines showed superior function under flooding situations. The soybean mutants would be valuable genetic resources to untie molecular mechanisms regulating soybean response to flood stress and numerous abiotic stress situations (Xiao et al., 2021). It is urgent to employ novel gene editing tools to develop flood-tolerant cultivars to counter the adverse effects of environmental changes. Base editing (BE) and prime editing (PE) could play a key role in speeding up the gene editing process in soybean. Several Cas proteins (Cas10, Cas12, and Cas13) are being used to edit the gene of interest in many crops. These crops can be used as a case study to expand the use of CRISPR/Cas9 in soybean. Large-scale use of CRISPR/Cas9 in soybean will help increase the area of soybean cultivation and counter the threats of abiotic stresses.

## Conclusions and future research direction

Flood stress significantly reduced soybean yield and quality and threatened food security. Soybean breeders are engaged in bringing genetic variation to breed flood-tolerant soybean cultivars. Soybean is extremely sensitive to flooding stress, and progress on genetic analysis of flood tolerance is insufficient to develop large number of flood-tolerant cultivars. The first and most important factor is genetic diversity which plays a key part in the acceleration of plant breeding schemes. We suggest preserving genetic diversity in future breeding programs is direly needed. Wild relatives have great potential to be used in conventional or molecular breeding; however, many techniques have been developed to develop flood tolerance in soybean, including conventional breeding methods (introduction, hybridization, and backcrossing), the use of hormones, and molecular breeding methods. Earlier investigations have been directed to examine hormonal effects in reducing the harmful effects of flood stress on soybean. Different plant hormones, ABA, ET, GA, IAA, and CK, have played a key role and improved soybean tolerance to flooding stress. However, the role of hormones has been deeply investigated; additional studies are obligatory to deeply explore the role of MT, CK, and GA.

QTL studies showed potent QTL, which control the flood tolerance in soybean. Several QTL were used in QTL pyramiding programs *via* marker-assisted selection; however, information about the success of these methods is limited. Most studies have suggested using the RIL population because of its advantage over other populations. GWAS-based QTL and gene identification paved the way for accelerating molecular breeding programs in soybean. The earlier gene pool would be an ideal source of genes for use in genetic engineering and CRISPR/Cas9. Genetic engineering is an ideal and powerful tool for developing transgenic soybean cultivars. Unfortunately, earlier work on genetically engineered soybean is not sufficient and more studies are needed to develop transgenic lines to maintain soybean growth on flooded soils. TFs and transcriptomes showed significant expression under flood stress, and these genetic factors could be edited by using CRISPR/Cas9. CRISPR/Cas9, a novel and influential gene manipulation tool, has been used in many crops to edit genes for abiotic stress tolerance and can be broadly used in soyeban. This review presented a detailed overview of different breeding techniques used to develop flood tolerance in soybean. This review will be an excellent source of informations for soybean breeders engaged in breeding against flood stress.

## Author contributions

Conceptualization, GJ and XZ. Writing—original draft preparation, GJ, ZQ, and AR. Writing—review and editing, MIH, IA, ZSH, MUH, MH, YM, YW, LC, WX, and WJ. All authors contributed to the article and approved the submitted version.
